# The Imaging Characteristics of Lens Subluxation on the Ultrasound Biomicroscopy

**DOI:** 10.1155/2022/7030866

**Published:** 2022-08-21

**Authors:** Aoxiang Wang, Dapeng Mou, Ningli Wang, Haiyan Wang

**Affiliations:** Beijing Tongren Eye Center, Beijing Tongren Hospital, Capital Medical University, Beijing Ophthalmology & Visual Sciences Key Lab, Beijing, China

## Abstract

**Background:**

To evaluate the imaging characteristics of the lens subluxation with the use of ultrasound biomicroscopy.

**Methods:**

From October 2018 to September 2019, 55 eyes diagnosed with lens subluxation were enrolled in the group. All patients underwent detailed eye examination and panoramic ultrasound biomicroscopy.

**Results:**

The most common sites of lens suspensory ligament injury were superior temporal side (32.73%) and superior nasal side (23.63%). The most common range of subluxation in all patients was 30°. Comparing the measurement indicators of all patients, ciliary body thickness (CBT) in affected eyes was smaller than that in healthy eyes (0.79 ± 0.21, 1.04 ± 0.16), the distance between ciliary process and crystal equator increased (1.91 ± 0.70, 1.17 ± 0.32), and iris-ciliary processes distance (ICPD) increased (1.04 ± 0.51, 0.80 ± 0.17) (*P* < 0.05). The range of subluxation in patients with lens subluxation was positively correlated with the distance between ciliary processes and the crystal equator.

**Conclusions:**

The ultrasound biological microscope has a good application significance in the diagnosis of lens subluxation. From this study, we suggest that the three indexes of CBT, ICPD, and the distance between the ciliary process and crystal equator are of high reference value in ultrasound biomicroscopy among patients with lens subluxation.

## 1. Introduction

Lens subluxation is a common ophthalmic disease, which refers to the change of lens position caused by a zonal abnormality. The causes of microzona abnormality and lens subluxation are varied, including ocular trauma, hereditary diseases (such as Marfan syndrome), and spontaneous subluxation. Global injury is the most common cause, accounting for 53%, while spontaneous subluxation is the rarest [1].

Ultrasound biomicroscopy (UBM) has unique advantages of being noninvasive and high-resolution in imaging of the anterior segment and intricate iridociliary complex with corneal haze or opacity [2, 3]. For example, it can provide visualization of the ciliary body and small zonal abnormalities that are not directly visible on slit-lamp examination. Pavlin [4] was the ﬁrst to describe the imaging of zonular ﬁbers used by 100 MHz UBM in the literature; after that, UBM has been widely used in observing the situation of zonule secondary to lens subluxation [5, 6]. This present study aimed to investigate the clinical and imaging features of lens subluxation in patients with the use of UBM.

## 2. Methods

### 2.1. Patients

A total of 52 patients (55 eyes) were enrolled in Beijing Tongren Hospital from October 2018 to September 2019, including 34 males and 18 females. The age of the selected patients was 30–81 years old, with an average age of (58.12 ± 14.0). Of the 55 eyes, 37 eyes had a history of ocular trauma (33 eyes with blunt trauma and 4 eyes with penetrating injury) and 18 eyes without any reason. There is a clear image of the anterior segment captured by UBM. Patients with open eyeball injury, congenital factors, iridocyclitis, and intraocular lens were excluded from this study.

### 2.2. Ophthalmic Examination

The ophthalmological examination included a review of medical history, measurement of best corrected visual acuity, measurement of intraocular pressure (Goldmann applanation tonometer), slit-lamp, and 50 MHz panoramic ultrasound biomicroscope (Sol Electronics Co., Ltd., model SW3200 L, China). UBM technology has been described before [6, 7]. In brief, a UBM examination was performed with the patient in a supine position in darkroom conditions using a 50-MHz transducer (Suoer Electronic Ltd., Model SW3200 L, China), and an experienced technician used a 2% methylcellulose eyecup and initially scanned over the central anterior chamber to observe for any tilt of the bright reﬂective line of the anterior lens capsule. Scanning was then performed over the iris root for 360° to assess the zonules directly. It was essential to ensure the long axis of the transducer was perpendicular to the zonular ﬁbers, which can be accomplished by having the patient position the eye accordingly or tilting the scanning probe appropriately. Efforts were made to ensure images provided a clear view of the scleral spur, angle, ciliary body, and a half-full chord of the iris.

### 2.3. UBM Imaging Quantitative Data

The UBM parameters in the current study have been defined by Pavlin et al. [8] and measured by the measurement tools built into the UBM machine (Figure 1). All linear parameters are measured in millimeters and angular parameters in degrees.

1. Anterior chamber depth (ACD): maximum distance from the inner surface of the cornea to the anterior surface of the lens. This parameter can directly reflect the degree of the anterior chamber.
2. Angle opening distance (AOD_500_): the distance between the corneal endothelial surface and the anterior surface of the iris measured on a line perpendicular to the trabecular meshwork at 500 *μ*m from the scleral spur. This parameter can reflect the degree of chamber angle opening indirectly.
3. Iris-ciliary processes distance (ICPD): the distance measured from the posterior surface of the iris to the ciliary process along the line extending from the corneal endothelium at 500 *μ*m from the scleral spur passing perpendicularly through the iris to the ciliary process.
4. Ciliary body thickness (CBT): the maximum thickness of the ciliary body truncated by a straight line perpendicular to the margin of the sclera. This parameter can reflect the state of regulation of the ciliary body.
5. Trabecular iris angle (TIA): to make a triangle with AOD 500 as the base and the recess at the iris root as the vertex, the included angle of the vertex was TIA. This parameter can reflect the degree of chamber angle opening indirectly.
6. Distance from the ciliary body to the equator of the lens: the distance between the point nearest the ciliary process to the lens and the equatorial terminal projection of the epithelial layer of the lens' anterior capsule.

### 2.4. Statistical Analysis

SPSS version 21.0 statistical software (SPSS, Inc., Chicago, IL) was used for data analysis. All UBM biometric data were expressed as mean ± standard deviation ($\bar{x}\pm s$). The probability value of *P* < 0.05 was considered to be statistically significant.

1. Comparisons of UBM parameters between lens subluxation eyes and contralateral eyes were performed with a *t*-test
2. The samples were divided into the trauma group and nontrauma group, and the related data were tested by the chi-square test.
3. Pearson correlation analysis was performed between lens subluxation range and other biometric values

### 2.5. Ethical Permission

The Ethics Committee of the Beijing Tongren Hospital (Beijing, China) approved the study procedure. The study adhered to the tenets of the Declaration of Helsinki and enrollment patients were provided with informed consent for the use of their medical records.

## 3. Results

### 3.1. Demographic and Clinical Characteristics

UBM scans of 55 eyes from 52 lens subluxation patients were analyzed. The mean age ± standard deviation (SD) of patients was 58.12 ± 14.00 years (30–81 years). There were more middle-aged and elderly patients aged 50–60 and 60–70, accounting for 28.85% and 23.08%, respectively. All patients had a large span of course time, ranging from 10 days to 50 years. Thirty-seven patients with a clear history of trauma were selected, whose course time centered on 1 week to 1 month and 1 month to 6 months, accounting for 27.03% and 32.43%, respectively.

All patients had poor naked visual acuity (55 eyes in total), and most patients were less than 20/60 (50 people, 90.91%). There were 26 patients (47.27%) with the best corrected visual acuity in the range of 20/200–20/60. 26 patients had cataract symptoms with different degrees. There were 16 patients with secondary glaucoma at the time of treatment, and some of them were using or had used intraocular pressure lowering (IOP) drugs. Therefore, the clinical reference value of intraocular pressure in this study is low, and the researchers did not provide detailed statistical data.

### 3.2. Comparative Analysis of UBM Imaging Quantitative Data

52 patients (55 eyes in total) were examined by UBM, and the range of lens subluxation was recorded (in clock code position). The criteria for determining lens subluxation and zonular abnormalities were as follows [4, 6]: (1) direct signs: rupture and elongation of the zonules. It is difficult to detect the line-like sound between the lens and ciliary body; (2) indirect signs: The ciliary body flattens at the junction or the equator of the lens becomes rounded and blunted. Zonular defect of 1 hour is the most common, with a total of 24 eyes, accounting for 43.64%; patients at 2 hours followed, a total of 15 eyes, accounting for 29.09%.

Fifty-two patients (103 eyes in total, including 1 patient with a contralateral prosthetic eye) underwent UBM, and general data on UBM biometric values are documented. *t*-test, *P* < 0.05 was statistically significant. The result shows that there was no significant difference in the measurement of AOD_500_ between the affected and healthy eyes; there were significant differences in ACD, CBT, distance from ciliary process to the equator of the lens, and ICPD. Among them, the differences between CBT and the distance from the ciliary process to the equatorial part of the lens were the most obvious; and subtle difference was found in TIA, i.e., the anterior chamber angle (Table 1).

The images of the center of subluxation in 55 eyes were intercepted. The biological eigenvalues of the center of the subluxation range and the corresponding cross-section were recorded and compared. The paired *t*-test was used to detect differences. *P* < 0.05 was statistically significant. The results showed that there was no significant difference in AOD_500_ and TIA. While, there were statistically significant differences in ciliary body thickness (CBT), the ciliary process to equatorial distance, and iris-ciliary body distance (ICPD) (Table 1).

The parameters of the center of the subluxation range of the affected eye and the corresponding parts of the healthy eye were recorded and the paired *t*-test was performed. *P* < 0.05 was considered statistically significant. Of all the metrics, only TIA was statistically significant (Table 1).

Spearman's rank correlation coefficient was performed to analyze the number of hours of subluxation recorded in 55 affected eyes and other biometric values. *P* < 0.05 indicated a statistically significant difference. The results showed that the number of hours of subluxation range was positively correlated with the distance of the ciliary process to the equatorial part of the lens (*P* < 0.05, correlation coefficient = 0.28) (Table 2).

Using the same measurement and statistical methods described above, data were recorded and analyzed in 37 eyes with a clear history of ocular trauma (Tables 3 and 4). *P* < 0.05 was considered statistically significant. In the comparison between the affected eye and the healthy eye, the results showed that there were statistically significant differences in CBT, the distance from the ciliary body to the lens equator, and the ICPD. The results of comparison between the center of the subluxation range and the corresponding cross-section in 37 eyes showed only the difference in TIA was statistically significant. The number of hours of subluxation was significantly correlated with the distance from the ciliary process to the equator of the lens (*P* < 0.05, correlation coefficient = 0.47).

## 4. Discussion

Accurate preoperative localization of the lens is necessary for treatment because most lens subluxation cases need surgery [5]. General clinical observation through slit-lamp examination found iris enlargement, vitreous prolapse, and partial quadrant lens subluxation; the diagnosis of obvious lens subluxation is not difficult. If the above signs are found in the slit-lamp examination, it is believed that the range of subluxation may be very large [9].

UBM is the only available examination for noninvasive, high-resolution imaging of anterior segment imaging due to its distinctive ability to image through corneal opacities [10]. Many types of research studies had demonstrated that UBM is of great value in identifying subclinical abnormalities of anterior segments, including slight lens subluxation, not easily visible on clinical exams, and may be invaluable in surgical planning and therapeutic management [3, 11, 12].

Our study confirmed that UBM can clearly visualize the status of the zonule and its surrounding anterior segments and measure relevant indicators. The results of this study also showed that CBT, the distance from the ciliary body to the equator of the lens, and ICPD had more reference valuable in lens subluxation patients with UBM examination. Affected eyes typically presented with a flattening of the ciliary body, reduced ciliary body thickness, increased ciliary process to the equatorial part of the lens, and increased ciliary body distance on UBM. There were statistically significant differences in the above three indicators between the affected eyes and the healthy eyes. Specifically, the thickness of the ciliary body in the affected eyes was smaller than that in the healthy eyes. There were significant differences in the above three indexes between the center of subluxation and the contralateral side of the same cross-section, indicating that CBT decreased and iris-ciliary body distance and ICPD increased. The results of the analysis of 37 eyes with clear ocular trauma were the same as the total of 55 eyes'. The possible reasons are as follows: (1) When the lens is subluxated, the lens equator of the subluxated side appears more curved than that of the side with an intact zonule [12]. The fracture or loss of zonule in the affected eye results in contraction and flattening of the internal muscle of the ciliary body and a smaller thickness than that of the healthy eye [13, 14]. (2) The slight abnormal function of the zonule leads to the change of lens position, which may be more obvious in the distance from ciliary process to the equator of lens and ICPD.

It is worth pointing out that one of the clinically common indexes to evaluate the lens' abnormal position, anterior chamber depth, showed less statistically significant differences in the UBM results of 37 affected eyes caused by trauma compared with healthy eyes. Lens subluxation is often suspected when asymmetric anterior chamber depth is observed [15]. However, for patients with ocular trauma, the factors are more complex. First of all, the source and direction of external force could impair the zonule to different degrees; second, the examination of anterior chamber depth is also affected by the examination position [12]. Therefore, during UBM, signs of shallow anterior chamber depth are difficult to detect in UBM imaging. Although the sign of the shallow depth of the anterior chamber can be used as the diagnostic guidance of slit-lamp examination, for patients with complex traumatic factors, special attention should be paid to negative symptoms, which cannot be used as a criterion for excluding the diagnosis of lens subluxation.

In this study, the researchers also conducted statistical analysis on the biometrics at the center of the range of subluxation and the corresponding site of the healthy eye and found that only the difference in TIA was statistically significant, no matter all 55 affected eyes or 37 eyes with ocular trauma. This may prompt us the zonule damage may have a greater impact on the ciliary body surrounding lesions than the relative structure of the opposite side, especially to the eyes with small range subluxation.

We examined the correlation between the range of lens subluxation, i.e., the number of hours of zonule defect and other biometric measurements of both affected eyes and traumatic eyes. The results indicated that the distance from the ciliary process to the equatorial part of the lens was longer when the lesion area of the zonule was larger. According to this result, we can conclude that the distance from the ciliary process to the equatorial part of the lens can be deemed as an index to judge the range of subluxations, regardless of whether the injury is accompanied by traumatic factors. It also indicates that the range of lens subluxation can be estimated by the distance from the ciliary process to the equatorial part of the lens. For UBM technicians, when you encounter a long distance from the ciliary process to the equator of the lens, you need to pay more attention to other relevant indicators to understand whether the patient has subluxation of the lens and to provide a more accurate and comprehensive imaging description. The same idea can be found in the study put forward by Noor A [16]. They have applied new methods in the study, and the conclusions drawn can also give some support to this study.

The measurement data in this study were mainly from patients with combined ocular trauma factors and nontraumatic factors, and patients with congenital abnormalities were not analyzed.

## 5. Conclusion

In summary, UBM can be used to diagnose and observe lens subluxation and to make up for the deficiency of slit-lamps and other examination methods. We concluded that the UBM of lens subluxation is characterized by a decrease in the thickness of the ciliary body, an increase in the distance from the ciliary body to the lens equator, and an increase in ICPD. The changes in the above three parameters have important reference values.

## Figures and Tables

**Figure 1:** Schematic diagram of measurement index. The red double arrow line is the measurement index line, and the white dotted line is the auxiliary line.

**Table 1:** UBM parameters comparison of total of 55 affected eyes.

	ACD (mm)	AOD_500_ (mm)	TIA (°)	CBT (mm)	Distance from the ciliary process to equator of the lens (mm)	ICPD (mm)
Affected eyes (55)	2.36 ± 0.97	0.41 ± 0.24	29.99 ± 13.81	0.79 ± 0.21	1.91 ± 0.70	1.04 ± 0.51
Healthy eyes (49)	2.61 ± 0.46	0.38 ± 0.14	33.41 ± 7.59	1.04 ± 0.16	1.17 ± 0.32	0.80 ± 0.17
*P*	0.04	0.29	0.05	0	0	0.003

The center of the subluxation range	2.36 ± 0.97	0.41 ± 0.24	29.51 ± 13.70	0.79 ± 0.21	1.91 ± 0.70	1.04 ± 0.51
The corresponding cross-section	—	0.36 ± 0.21	28.69 ± 10.43	1.10 ± 0.33	1.17 ± 0.45	0.73 ± 0.51
*P*	—	0.1	0.54	0	0	0

The cross-section of the center of the subluxation range of the affected eye	0.36 ± 0.21	28.69 ± 10.42	1.10 ± 0.33	1.17 ± 0.45	0.73 ± 0.51	0.36 ± 0.21
The corresponding place of the healthy eyes	0.37 ± 0.12	32.50 ± 6.11	1.92 ± 0.21	1.18 ± 0.55	0.79 ± 0.45	0.37 ± 0.12
*P*	0.68	0	0.19	0.81	0.45	0.68

**Table 2:** Correlation analysis between the number of hours of subluxation and UBM parameters in a total of 55 affected eyes.

	Correlation coefficient	*P*
Number of hours of subluxation, ACD	0.18	0.20
Number of hours of subluxation, AOD_500_	0.10	0.48
Number of hours of subluxation, TIA	0.15	0.26
Number of hours of subluxation, CBT	−0.09	0.51
Number of hours of subluxation, the distance from the ciliary process to the equator of the lens	0.28	0.03
Number of hours of subluxation, ICPD	0.11	0.44

**Table 3:** UBM parameters comparison of 37 eyes with ocular trauma.

	ACD (mm)	AOD_500_ (mm)	TIA (°)	CBT (mm)	Distance from ciliary process to equator of the lens (mm)	ICPD (mm)
Affected and healthy eyes						
Affected eyes (37)	2.29 ± 1.00	0.464 ± 0.052	29.54 ± 14.12	0.77 ± 0.19	1.99 ± 0.75	1.05 ± 0.53
Healthy eyes (37)	2.57 ± 0.45	0.409 ± 0.028	33.69 ± 638	1.05 ± 0.17	1.07 ± 0.26	0.81 ± 0.14
*P*	0.67	0.36	0.07	0	0	0.02

The center of the subluxation range and the corresponding cross-section in the affected eyes						
The center of the subluxation range	2.29 ± 1.00	0.40 ± 0.26	28.41 ± 13.81	0.76 ± 0.18	2.08 ± 0.69	1.04 ± 0.50
The corresponding cross-section	—	0.32 ± 0.17	27.09 ± 8.96	1.11 ± 0.32	1.12 ± 0.42	0.80 ± 0.54
*P*	—	0.21	0.45	0	0	0.02

The cross-section of the center of the subluxation range of the affected eye and the corresponding place of the healthy eyes						
The cross-section of the center of the subluxation range of the affected eye	0.34 ± 0.18	27.81 ± 9.38	1.07 ± 0.33	1.08 ± 0.43	0.78 ± 0.57	0.34 ± 0.18
The corresponding place of the healthy eyes	0.38 ± 0.13	33.80 ± 6.45	1.05 ± 0.17	1.07 ± 0.26	0.80 ± 0.14	0.38 ± 0.13
*P*	0.14	0	0.82	0.85	0.82	0.138

**Table 4:** Correlation analysis between the number of hours of subluxation and UBM parameters in 37 eyes with traumatic factor.

	Correlation coefficient	*P*
Number of hours of subluxation, ACD	0.10	0.56
Number of hours of subluxation, AOD_500_	0.14	0.43
Number of hours of subluxation, TIA	0.15	0.39
Number of hours of subluxation, CBT	−0.19	0.25
Number of hours of subluxation, the distance from the ciliary process to the equator of the lens	0.47	0.00
Number of hours of subluxation, ICPD	0.22	0.20

## Data Availability

The datasets used and analyzed during the current study are available from the corresponding author upon request.
